The article "Antistroke Network Pharmacological Prediction of Xiaoshuan Tongluo Recipe Based on Drug-Target Interaction Based on Deep Learning" was published in 2022. Journal: Comput Math Methods Med.

# Antistroke Network Pharmacological Prediction of Xiaoshuan Tongluo Recipe Based on Drug-Target Interaction Based on Deep Learning

**DOI:** 10.1155/2022/6095964

**Published:** 2022-08-02

**Authors:** Yongfu Zhou

**Affiliations:** School of Chemistry and Pharmaceutical Engineering Chongqing Industry Polytechnic College, Chongqing 401120, China

## Abstract

Stroke is a common cerebrovascular disease that threatens human health, and the search for therapeutic drugs is the key to treatment. New drug discovery was driven by many accidental factors in the early stage. With the deepening of research, disease-related target discovery and computer-aided drug design constitute a more rational drug discovery process. The deep learning model was constructed by using recurrent neural network, and then, the classification and prediction of compound-protein interactions were studied. In this study, the network pharmacological prediction of stroke based on deep learning is obtained. (1) In the case of discrete time, a distributed optimization algorithm with finite time convergence is applied. A distributed exact first-order algorithm for the case where the objective function is smooth. On the basis of the DGD algorithm, an additional cumulative correction term is added to correct the error caused by the fixed step size of DGD. Solve multiple optimization problems with equality constraints by using Lagrangian functions. Alternately update the original variable and the dual variable to get the solution of a large global problem. It converges to the optimal solution in an asymptotic or exponential way; that is, the node can reach the optimal solution more accurately when the time tends to infinity. (2) Deep learning, also sometimes called representation learning, has a set of algorithms that can automatically discover the desired classification or detection by feeding it into a machine using raw datasets. Multiple levels of abstraction are abstracted through the use of nonlinear models. This simplifies finding solutions to complex and nonlinear functions. Based on the automatic learning function, it provides the functions of modularization and transfer learning. Deep architectures, which usually contain hidden layers, differ from traditional machine learning, which requires a large amount of data to train the network. There are many levels of modules that are nonlinear and transform the information present on the first level into higher levels which are more abstract in nature and are basically used for feature extraction and transformation. (3) The accuracy rate of the framework based on the multitask deep learning algorithm is 91.73%, and the recall rate reaches 96.13%. The final model was predicted and analyzed using real sample data. In the inference problem, it has the advantages of fast training and low cost; in the generation problem, it also has the advantages of fast training, high stability, high diversity, and high quality of image reconstruction.

## 1. Introduction

Stroke, commonly known as “stroke,” is a common type of cerebrovascular disease that threatens human health. It has the characteristics of high morbidity, high mortality, high disability rate, and high recurrence rate. After stroke, the cortical swallowing center is damaged, namely, pseudobulbar palsy, which mainly affects the first two phases of the swallowing process—oral preparation phase and oral phase. Damage to the cortical swallowing center will cause severe swallowing disorders, and it will be impossible to control the swallowing intensity. Strokes are mostly due to internal injury accumulation, coupled with loss of work and rest, depression, uncontrolled diet, or invasion of external pathogens, resulting in the imbalance of yin and yang of the internal organs of the human body. Qi machine disorder, internal movement of liver wind, phlegm fire, channeling meridians, blocking the mind orifices, and thus sudden syncope eventually lead to brain tissue death; that is, the proportion of ischemic stroke is as high as 80%. Stroke disorders, including inhibitory neuronal circuits, will also be affected. The medulla oblongata swallowing center is damaged, that is, true bulbar palsy. After trauma to the medulla oblongata swallowing center, there will be abnormalities in the pharyngeal stage, pharyngeal muscle paralysis, levator laryngeal muscle weakness, pharyngeal dyskinesia, tongue muscle tremor, atrophy, slurred speech, prolonged swallowing reflex initiation, and difficulty swallowing. Food retention in the pharynx can easily cause asphyxia. Decreased input of sensory information will result in a delay in the initiation of swallowing, resulting in dysphagia. Stroke may cause extensive brain tissue damage leading to cognitive impairment. In inflammatory mechanism, cerebral ischemia causes blood-brain barrier diffusion dysfunction, inflammatory reaction, edema of brain cells, and neuronal death under the action of cytokines, chemokines, and reactive oxygen species. For the changes in neurotransmitter levels, when the levels of neurotransmitters associated with cognition are abnormal after stroke, cognitive impairment can also be caused. Abnormal levels of dopamine can lead to executive control impairment. Visual-spatial attention and working memory are innervated by cholinergic and dopaminergic pathways involving frontoparietal and frontostriatal networks [1–3]. Application of traditional Chinese medicine and acupuncture in the treatment of phlegm and blood stasis blocking collaterals type arrhythmia, to resolve phlegm and dissipate stagnation, Salvia, Dilong to promote blood circulation to remove blood stasis and dredging collaterals, licorice tablets to detoxify and reconcile various medicines, the whole formula clears phlegm and opens orifices, activates blood and dredges collaterals. The results show that Ditan Decoction combined with acupuncture in the treatment of poststroke dysphagia patients with phlegm and blood stasis blocking collaterals can effectively reduce the symptoms of dysphagia and the risk of aspiration and significantly reduce complications. As one of the complications after stroke, swallowing dysfunction has no specific name in ancient Chinese medicine books, but it is based on the causes of swallowing dysfunction (esophageal disease, throat disease, cerebrovascular accident, etc.). Traditional Chinese medicine decoction is a common treatment method in traditional Chinese medicine. Because of its advantages of simple preparation and rapid curative effect, it is often used for the treatment of dysphagia after stroke. The patients were treated with Bushen-Liyan Decoction and their symptoms were evaluated. The results showed that the total effective rate was 83.33% [4–6]. Qiyan Decoction can effectively treat patients with dysphagia after stroke with internal obstruction of blood stasis. This method is effective and safe. Acupuncture provides valuable practical experience in the treatment of dysphagia after stroke. Whether the swallowing function is normal or not is related to the tongue, pharynx, larynx, and other parts. Therefore, from the perspective of TCM meridians, swallowing function is related to the Ren meridian, the spleen meridian of the foot Taiyin, the stomach meridian of the foot Yangming, the kidney meridian of the foot Shaoyin, and foot Jueyin liver meridian. Acupuncture and moxibustion can effectively regulate the brainstem neuron network and the higher cortical center, make the cerebral cortex more active, restore the normal blood supply to the brain, and improve the level of central nervous system function; in addition, it can also allow the normal activities of the swallowing muscles. The research data of acupuncture treatment of poststroke dysphagia patients were collected and sorted, and a meta-analysis was carried out on this basis. The results showed that this treatment can improve the level of swallowing function. When dealing with a neural network, a loss function is preset, and then, an optimization algorithm can be used to minimize the loss value of the loss function. In the optimization algorithm, the set loss function is generally called the objective function of the optimization problem. Even if the optimization algorithm is used, it may not be guaranteed that all neural networks have good generalization errors. Therefore, in the process of neural network training, it is necessary to pay attention to problems such as overfitting and underfitting, so as to obtain the numerical solution of the objective function. It is necessary to choose suitable values to update the independent variables in the reverse direction along the gradient to reduce the value of the objective function. KEGG pathway enrichment of signaling pathways describe gene regulation [7–9]. Deep learning techniques define and design model inputs according to some principles, such as data packets, PCAP files, and flow statistical feature files. Second, models and algorithms are purposefully selected according to the features of the model and the purpose of the classifier. Finally, a deep learning classifier is trained to associate the inputs with the corresponding class labels. The training of deep learning models requires a large number of labeled samples, which are difficult to collect in real network environments. A flow feature extraction algorithm based on the concept of bidirectional flow is used to preprocess the malicious traffic dataset. It solves the problem of low recognition accuracy of traditional feature extraction algorithms and proposes a multitask-based deep learning model, which is more efficient than the single-task-based deep learning model on the public CIC-IDS2017 dataset and CIC-DDoS2019 dataset. For better performance, a data preprocessing scheme was proposed to construct a feature extraction algorithm based on the concept of bidirectional flow and a malicious traffic monitoring system with a multitask deep learning CNN model. The experiment is a subset of the public CIC-IDS2017 dataset and the CIC-DDoS2019 dataset. The malicious traffic of some malicious traffic categories in all the datasets is less than the malicious traffic of the malicious traffic category selected in this paper [10–12]. Class imbalance is an important problem in malicious traffic classification, and how to eliminate the training impact brought by this class imbalance is a valuable research in the future. In the multitask-based deep learning training experiment, we found that if the loss weights of different tasks are correctly combined for the three tasks, the accuracy of each task recognition is also different. So how to set the most appropriate combination of loss weights to achieve the best learning accuracy is a valuable research. There are only a dozen types of malicious traffic identified by the malicious traffic monitoring system based on multitask deep learning, so capturing and collecting enough malicious traffic types is an important part of our next work. The deep learning model was constructed by using recurrent neural network, and then, the classification and prediction of compound-protein interactions were studied. Complete the collection and preprocessing of experimental data. Postconditions are related to the initial and final states, assuming that all other threads obey the dependency constraints [13–15]. The key to achieving compositionality is to reformulate interference-free tests.

## 2. Drug Target Prediction

### 2.1. Predicting Drug-Target Interactions

“Drug discovery,” as a research direction at the intersection of biology, chemistry, and informatics, represents the unremitting efforts of human beings to contribute to survival and health. As shown in Figure 1, drug discovery was driven by many accidental factors in the early stage. With the deepening of research, the two links of disease-related target discovery and computer-aided drug design together constitute a more rational drug discovery process. Systems pharmacology is derived from presystems biology and emphasizes the integration of multilevel and multiomics information. The latter is often compared to the “design key,” which takes structural biology and analytical chemistry as the source of thought, and derives structure-based drug design, usually referring to LBDD with clear binding site structure information and ligand-based drug design. Traditional drug discovery mostly follows the assumption of “single target-local antagonism”; that is, it is assumed that the mechanism of action of a drug is that a certain single component acts on a certain single target, and then through the downstream signaling pathway, and finally affects the phenotype, that is, from the drug molecule to the phenotype. From molecular target to final phenotype, it goes through a linear “mechanical process.” Such assumptions have profoundly affected the whole process of drug discovery from methodology and preclinical research system to clinical trial design, including computer-aided drug design usually targeting a certain target or binding site; research based on systems pharmacology or network medicine is often attributed to finding a molecule that conforms to the characteristics of the network structure or a molecule on the core link of the key mechanism as a target.

### 2.2. Drug-Disease Relationship Prediction Algorithm

Under the assumption of low rank, the bounded kernel norm regularization method (BNNR) was used to complete the drug-disease matrix. BNNR is performed on adjacency matrices of heterogeneous drug-disease networks integrating drug-drug, drug-disease, and disease-disease networks. But integrating all similar networks can introduce noise into the data, as shown in Figure 2. Matrix factorization and matrix completion techniques have been applied to drug relocalization in recent years. Including the interaction network among genes, a matrix decomposition model was established. Using the information in the gene network, the relationship between drugs and diseases can be predicted, and new indications of known drugs can be obtained. The drug-drug relationship network, disease-disease relationship network, and drug-disease relationship network were integrated to construct a heterogeneous network, and then, the dominant singular value and the corresponding singular vector of the association matrix were efficiently calculated using R4SVD. Based on the singular value threshold (SVT) algorithm, a drug relocation recommendation system (DRRS) is proposed to rank the potential associations between drugs and diseases by complementing the drug-disease association matrix. The loss function, also known as the cost function, is used as a learning criterion for optimizing the parameters of the neural network. The loss function is used to measure the degree of difference between the predicted value of the model and the real value. It is a nonnegative real-valued function. The better the model fits the real value, the smaller the loss function. The worse the model fits the true value, the larger the value of the loss function. Similar to the choice of activation function, the types of loss functions used by different models and problems are also different. The loss functions are generally divided into empirical risk loss functions and structural risk loss functions.

## 3. Deep Learning Algorithms

### 3.1. LDAP [16–20]

(1) $$\begin{array}{c} \min f\left(x\right)+g\left(z\right). \end{array}$$

Classifier:

(2) $$\begin{array}{c} \text{s}.\text{t}.Ax+Bz=c,\\ p^{*}=\inf\left\{f\left(x\right)+g\left(z\right)\left|Ax+Bz=c\right.\right\}. \end{array}$$

Marked samples:

(3) $$\begin{array}{c} L_{\rho }\left(x,y,z\right)=f\left(x\right)+g\left(z\right)+y^{T}\left(Ax+Bz-c\right)+\frac{\rho }{2}{\left\|Ax+Bz-c\right\|}_{2}^{2},\\ x^{k+1}=\arg\underset{x}{\min}L_{p}\left(x,z^{k},y^{k}\right). \end{array}$$

Dataset:

(4) $$\begin{array}{c} z^{k+1}=\arg\underset{z}{\min}L_{p}\left(x^{k+1},z,y^{k}\right),\\ y^{k+1}=y^{k}+\rho \left({Ax}^{k+1}+{Bz}^{k+1}-c\right). \end{array}$$

### 3.2. NSSQL [21–23]

Feature extraction algorithm for bidirectional flow concept:

(5) $$\begin{array}{c} \overset{n}{\underset{i=1}{\sum }}f_{i}\left(x\right)+g\left(x\right). \end{array}$$

Loss function:

(6) $$\begin{array}{c} \min\overset{n}{\underset{i=1}{\sum }}f_{i}\left(x_{i}\right)+g\left(z\right)\\ \text{s}.\text{t}.x_{i}-z=0,i=1,\cdots ,n. \end{array}$$

Multitask deep learning:

(7) $$\begin{array}{c} L_{\rho }\left(\left\{x_{i}\right\},z,\left\{y_{i}\right\}\right)=\overset{n}{\underset{i=1}{\sum }}\left(f{\left(x_{i}\right)}_{i}+y_{i}^{T}\left(x_{i}-z\right)+\frac{\rho }{2}{\left\|x_{i}-z\right\|}_{2}^{2}\right)+g\left(z\right). \end{array}$$

Monitoring system identification:

(8) $$\begin{array}{c} x_{i}^{k+1}=\arg\min f_{i}{\left(x_{i}\right)}_{i}+y_{i}^{kT}\left(x_{i}-z^{k}\right)+\frac{\rho }{2}{\left\|x_{i}-z^{k}\right\|}_{2}^{2},\\ z^{k+1}=\arg\min\left(g\left(z\right)+\overset{n}{\underset{i=1}{\sum }}\left(-y_{i}^{kT}z+\frac{\rho }{2}{\left\|x_{i}^{k+1}-z\right\|}_{2}^{2}\right)\right). \end{array}$$

Compound-protein interactions:

(9) $$\begin{array}{c} y_{i}^{k+1}=y_{i}^{k}+\rho \left(x_{i}^{k+1}-z^{k+1}\right). \end{array}$$

Activation function:

(10) $$\begin{array}{c} \min\overset{n}{\underset{i=1}{\sum }}f_{i}\left(x_{i}\right)+g\left(\overset{n}{\underset{i=1}{\sum }}x_{i}\right). \end{array}$$

Multiomics information integration:

(11) $$\begin{array}{c} L_{\rho }\left(\left\{x_{i}\right\},\left\{z_{i}\right\},\left\{y_{i}\right\}\right)=\overset{n}{\underset{i=1}{\sum }}\left(f_{i}{\left(x_{i}\right)}_{i}+y_{i}^{T}\left(x_{i}-z_{i}\right)+\frac{\rho }{2}{\left\|x_{i}-z_{i}\right\|}_{2}^{2}\right)+g\left(\overset{n}{\underset{i=1}{\sum }}z_{i}\right). \end{array}$$

### 3.3. NetBIOS [24–26]

Systems pharmacology:

(12) $$\begin{array}{c} x_{i}^{k+1}=\arg\min\left(f_{i}\left(x_{i}\right)+\frac{\rho }{2}{\left\|x_{i}-z_{i}^{k}+u_{i}^{k}\right\|}_{2}^{2}\right),\\ z_{i}^{k+1}=\arg\min\left(g\left(\overset{n}{\underset{i=1}{\sum }}z_{i}\right)+\overset{n}{\underset{i=1}{\sum }}\left(\frac{\rho }{2}{\left\|z_{i}-x_{i}^{k}-u_{i}^{k}\right\|}_{2}^{2}\right)\right). \end{array}$$

Single target:

(13) $$\begin{array}{c} u_{i}^{k+1}=u_{i}^{k}+x_{i}^{k+1}-z_{i}^{k+1},\\ \min g\left(n\bar{z}\right)+\frac{\rho }{2}\left(\overset{n}{\underset{i=1}{\sum }}{\left\|z_{i}-\alpha_{i}\right\|}_{2}^{2}\right). \end{array}$$

Downstream signaling pathway:

(14) $$\begin{array}{c} \bar{z}=\frac{1}{n}\overset{n}{\underset{i=1}{\sum }}z_{i}. \end{array}$$

Molecular target:

(15) $$\begin{array}{c} x_{i}^{k+1}=\arg\min\left(f_{i}\left(x_{i}\right)+\frac{\rho }{2}{\left\|x_{i}-x_{i}^{k}+{\bar{x}}^{k}-{\bar{z}}^{k}+u^{k}\right\|}_{2}^{2}\right). \end{array}$$

Regularization method:

(16) $$\begin{array}{c} z^{k+1}=\arg\min\left(g\left(n\bar{z}\right)+\frac{n\rho }{2}{\left\|\bar{z}-x^{k+1}-u^{k}\right\|}_{2}^{2}\right). \end{array}$$

Drug-disease matrix:

(17) $$\begin{array}{c} s\left(i,j\right)=\left(X*W\right)\left(i,j\right)=\underset{m}{\sum }\underset{n}{\sum }x\left(i+m,j+n\right)w\left(m,n\right). \end{array}$$

Predicting drug-disease relationships:

(18) $$\begin{array}{c} \min\overset{n}{\underset{i=1}{\sum }}f_{i}\left(w_{i}\right)+g\left(w\right),\\ \min\overset{n}{\underset{i=1}{\sum }}f_{i}\left(w_{i}\right)+\frac{\lambda }{2}{\left\|w_{i}-w\right\|}^{2}. \end{array}$$

## 4. Simulation Experiment

### 4.1. Distributed Algorithm

The ADMM algorithm can decompose a complex problem into a simple subproblem, so as to solve the problem in parallel. Early distributed optimization algorithms were distributed subgradient algorithms. DGD is a simple distributed first-order gradient descent algorithm suitable for solving nonsmooth convex functions. Distributed optimization algorithms that converge in finite time can be divided into discrete and continuous. In the discrete-time case, a distributed optimization algorithm with finite-time convergence is applied. Each agent performs its own consensus step and then descends along the local subgradient of its own convex objective function. As shown in Table 1 and Figure 3, the experimental results are shown in data 1, Accu.(%) = 41.43, Prec.(%) = 59.13, Sen.(%) = 48.04, MCC (%) = 73.83, and AUC (%) = 72.12. But this algorithm only works for balanced graphs. In dataset 6, Accu.(%) = 65.15, Prec.(%) = 68.77, Sen.(%) = 77.3, MCC (%) = 62.52, and AUC (%) = 75.77.

### 4.2. ADMM General Form

It is shown in Table 2 and Figure 4. The problem of selectivity and invariance is the main difficulty of conventional machine learning; therefore, the ability of these methods to deal with data in raw form is limited. In the LDAP category, BF − Alg Accu = 82.4, BF − Alg Recall = 97.31, BF − Alg F1 − score = 87.86, T − Alg Accu = 98.82, T − Alg Recall = 90.21, and T − Alg F1 − score = 81.15. Each layer takes the output of the previous layer as input and applies nonlinear transformations to extract useful features for classification. Selectivity versus invariance means selecting those features that contain more information and ignoring those features that contain less information about the parameters; i.e., the selected features should be different from each other. In the TFTP category, BF − Alg Accu = 95.94, BF − Alg Recall = 87.95, BF − Alg F1 − score = 90.74, T − Alg Accu = 83.91, T − Alg Recall = 98.53, and T − Alg F1 − score = 98.91. Deep learning, sometimes called representation learning, has a set of algorithms that can automatically discover desired classifications or detections by feeding them into machines using raw datasets. Deep learning methods abstract multiple levels of abstraction by using nonlinear models. This simplifies finding solutions to complex and nonlinear functions. Deep learning is based on the automatic learning function and provides the function of modularization and transfer learning. Deep learning usually includes deep architectures with hidden layers, and unlike traditional machine learning, deep learning requires a large amount of data to train the network. There are many levels of modules in deep learning which are nonlinear and transform the information present on the first level into higher upper levels which are more abstract in nature and are basically used for feature extraction and transformation.

### 4.3. Autoencoders

The encoder operation converts the input vector into a compressed representation, while the decoder operation attempts to reconstruct from input variables. The sizes of the input and output layers are equal, and the size of the hidden layer must be smaller than the size of the input layer. The acquired information will inevitably contain a lot of noise, or the information is very rich and diverse. Whether it is noise information or other information irrelevant to the subsequent tasks, it is not helpful for subsequent tasks such as classification and recognition. The dimension of the original data feature space is reduced to obtain a set of classification samples with low probability of classification error and no redundancy. The scale of data information grows very fast, and linear discriminant analysis, autoencoder, isometric mapping, local linear embedding, and traditional autoencoders have developed many improved models based on autoencoders through continuous development. As shown in Table 3 and Figure 5, the tuning results are F1 − score = 92.12, Accuracy = 80.92, AUC = 95.23, AUPR = 84.94, Loss = 96.49, Precision = 95.19, Recall = 97.54, and Specificity = 83.33. Since the vector output by the traditional autoencoder is unknown and disordered, the autoencoder can only learn data but cannot actively generate data. At the same time, the feature vector of the hidden layer lacks continuity, that is, under small disturbances, the generated data will be very strange and very deviating from the input data of the original model. The hidden layer obtained in the traditional autoencoder coding network is changed to obtain the mean and variance, and then, from the normal distribution satisfying the mean and variance, the mean and variance are uniquely determined. The output of both the encoder and the decoder in the variational autoencoder are probability density distributions, and the variables in the probability distribution are constrained by parameters. For common data such as pictures, videos, and audios, it is often assumed that they are generated by some lower-level variables, and these variables satisfy some specific distributions, which are called latent variables or latent variables. These hidden variables represent the internal structure of the data or some kind of abstraction. In order to solve the inference problem, the main methods are Monte Carlo Markov chain and variational inference. Because Monte Carlo Markov chains require large batches of data at each step in training, the training cost is very high. Compared with the inference problem, it has the advantages of fast training and low cost. In the generation problem, it also has the advantages of fast training, high stability, high diversity, and high image reconstruction quality. The disadvantages are low definition and so on.

### 4.4. Deep Learning Model Training

Its input is preserved due to the deep learning modulo internal memory. Just like human behavior, it takes into account the information it currently has as well as previous experience gained through loops when making a decision. The most popular implementation is long short-term memory, which backpropagates errors through layers, learning in a circular fashion. According to these characteristics of network traffic, identification techniques in data mining can be used to achieve good traffic identification through machine learning. In network traffic identification, this prior knowledge can be different characteristics of network traffic and personnel supervision information. Choosing an appropriate machine learning algorithm can make full use of prior knowledge to complete traffic identification. As shown in Table 4 and Figure 6, in DNN EDTPs1 prediction, Dataset = 3216, Recall (0.9) = 13.62, Samplesa = 18, and Recall (0.5) = 40.67. When the traffic characteristics are easily outdated quickly, there are many observation samples, and the learning efficiency is not very high. A framework based on multitask deep learning algorithms is included. Separate and purify the PCAP files of the public datasets according to traffic categories. In view of the fact that the packets are captured at the link layer, some data packets may be ARP protocol, etc., and there is no upper layer information, so these data packets are regarded as invalid packets. In addition, some data packets have no port information, and an exception will be thrown. These packets are discarded. Using timestamp, source ip, source port, destination ip, and destination port, the data packets of the PCAP file are purified into a new PCAP file according to the malicious traffic type according to the collection information of malicious traffic. The prediction results of SVM EDTPs1 are Dataset = 3216, Recall (0.9) = 32.19, Samplesa = 17, and Recall (0.5) = 58.06. The data fed into the model training needs to be detected outliers; otherwise, the recognition performance of the model may be degraded. The outliers in the flow features are eliminated and normalized. The label data needs to be labeled according to the classification rules of the task to form a label file with the same sample size as the dataset. It also helps the classification task to converge faster during model training after the label file is formed. The dataset is divided into three parts before model training, which are used as the input of the main task, auxiliary task, and model test, respectively; after the model is constructed, the test data is used to test the model, and finally, the three parts of the multitask deep learning model are output. Each task recognition result outputs the confusion matrix of the main task and four performance evaluation indicators: precision, recall, F1-Score and accuracy.

## 5. Conclusion

Stroke is a common cerebrovascular disease that threatens human health, and the search for therapeutic drugs is the key to treatment. New drug discovery is driven by many accidental factors in the early stage. With the deepening of research, the two links of disease-related target discovery and computer-aided drug design together constitute a more rational drug discovery process. The deep learning model was constructed by using recurrent neural network, and then, the classification and prediction of compound-protein interactions were studied. Complete the collection and preprocessing of experimental data. Postconditions are related to the initial and final states, assuming that all other threads obey the dependency constraints. The key to achieving compositionality is to reformulate interference-free tests. (1) In the discrete-time case, a distributed optimization algorithm with finite-time convergence is applied. Each agent performs its own consensus step and then descends along the local subgradient of its own convex objective function. Under the assumption that the subgradient is bounded, the distributed subgradient descent algorithm with gradually decreasing step size can gradually converge to a domain of the optimal solution. When the objective function is smooth, a distributed exact first-order algorithm can be obtained. The central idea is to add an additional cumulative correction term based on the DGD algorithm to correct the error caused by the fixed step size of DGD. The experimental results are shown in data 1, Accu.(%) = 41.43, Prec.(%) = 59.13, Sen.(%) = 48.04, MCC (%) = 73.83, and AUC (%) = 72.12. But this algorithm only works for balanced graphs. It is allowed to use its local continuous state arbitrarily to obtain the optimal value within a limited time step. The optimal value is obtained when the network topology graph is a directed graph and is strongly connected. Alternating direction multiplier method is to solve multiple optimization problems with equality constraints through Lagrangian functions. Alternately update the original variable and the dual variable to get the solution of a large global problem. In dataset 6, Accu.(%) = 65.15, Prec.(%) = 68.77, Sen.(%) = 77.3, MCC (%) = 62.52, and AUC (%) = 75.77. Most of the algorithms converge to the optimal solution in an asymptotic or exponential manner, that is, the nodes can reach the optimal solution more accurately when the time tends to infinity. (2) The problem of selectivity and invariance is the main difficulty of conventional machine learning; therefore, the ability of these methods to deal with data in raw form is limited. In the LDAP category, BF − Alg Accu = 82.4, BF − Alg Recall = 97.31, BF − Alg F1 − score = 87.86, T − Alg Accu = 98.82, T − Alg Recall = 90.21, and T − Alg F1 − score = 81.15. Each layer takes the output of the previous layer as input and applies nonlinear transformations to extract useful features for classification. Selectivity versus invariance means selecting those features that contain more information and ignoring those features that contain less information about the parameters; i.e., the selected features should be different from each other. In the TFTP category, BF − Alg Accu = 95.94, BF − Alg Recall = 87.95, BF − Alg F1 − score = 90.74, T − Alg Accu = 83.91, T − Alg Recall = 98.53, and T − Alg F1 − score = 98.91. (3) Traditional autoencoders such as autoencoder, isometric mapping, and local linear embedding have been developed continuously, and many models based on autoencoder improvement have been developed. As shown in Table 3 and Figure 5, the tuning results are F1 − score = 92.12, Accuracy = 80.92, AUC = 95.23, AUPR = 84.94, Loss = 96.49, Precision = 95.19, Recall = 97.54, and Specificity = 83.33. Since the vector output by the traditional autoencoder is unknown and disordered, the autoencoder can only learn data but cannot actively generate data. At the same time, the feature vector of the hidden layer lacks continuity; that is, under small disturbances, the generated data will be very strange and very deviating from the input data of the original model. (4) Selecting an appropriate machine learning algorithm can make full use of prior knowledge to complete traffic identification. As shown in Table 4 and Figure 6, in DNN EDTPs1 prediction, Dataset = 3216, Recall (0.9) = 13.62, Samplesa = 18, and Recall (0.5) = 40.67. When the traffic characteristics are easily outdated quickly, there are many observation samples, and the learning efficiency is not very high. A framework based on multitask deep learning algorithms is included. Separate and purify the PCAP files of the public datasets according to traffic categories. The prediction results of SVM EDTPs1 are Dataset = 3216, Recall (0.9) = 32.19, Samplesa = 17, and Recall (0.5) = 58.06.

## Figures and Tables

**Figure 1:** Schematic diagram of network target.

**Figure 2:** Distributed learning framework.

**Figure 3:** The experimental results of the autoencoder.

**Figure 4:** Model performance comparison.

**Figure 5:** The experimental results of network parameter tuning.

**Figure 6:** Classification model prediction results.

**Table 1:** Experimental results of autoencoder.

Test set	Accu. (%)	Prec. (%)	Sen. (%)	MCC (%)	AUC (%)
1	41.43	59.13	48.04	73.83	72.12
2	42.82	85.9	43.96	66.69	75.94
3	61.88	60.22	84.56	70.2	88.81
4	74.26	43.75	82.02	83.36	86.93
5	75.39	63.51	49.35	51.89	83.8
6	65.15	68.77	77.3	62.52	75.77

**Table 2:** Model performance comparison.

	BF-Alg Accu	BF-Alg Recall	BF-Alg F1-score	T-Alg Accu	T-Alg Recall	T-Alg F1-score
LDAP	82.4	97.31	87.86	98.82	90.21	81.15
NSSQL	91.11	82.53	88.61	86.47	96.25	90.91
NetBIOS	96.61	89.38	92.28	98.08	82.48	82.75
SYN	84.95	85.93	90.61	82.83	92.77	97.04
TFTP	95.94	87.95	90.74	83.91	98.53	98.91

**Table 3:** Experimental results of network parameter tuning.

	2	3	4
F1-score	92.12	82.43	88.56
Accuracy	80.92	85.27	91.06
AUC	95.23	86.24	93.88
AUPR	84.94	98.92	88.93
Loss	96.49	89.19	95.65
Precision	95.19	85.07	82.03
Recall	97.54	86.09	93.03
Specificity	83.33	80.4	89.41

**Table 4:** Model prediction results.

Method	Dataset	Recall (0.9)	Samplesa	Recall (0.5)
DNN EDTPs1	3216	13.62	18	40.67
DNN EDTPs2	3827	9.09	14	71.98
DNN EDTPs	7043	23.46	14	88.36
HN EDTPs1	3216	21.89	17	76.88
HN EDTPs2	3827	31.59	19	58.29
HN EDTPs	7043	12.37	19	55.39
RNN EDTPs1	3216	24.64	20	43.58
RNN EDTPs2	3827	45.67	17	46
RNN EDTPs	7043	14.54	10	52.5
RF EDTPs1	3216	24.79	15	47.17
RF EDTPs2	3827	24.8	16	47.84
RF EDTPs	7043	25.44	17	81.09
SVM EDTPs1	3216	32.19	17	58.06
SVM EDTPs2	3827	31.76	18	59.54
SVM EDTPs	7043	37	13	67.21

## Data Availability

The experimental data used to support the findings of this study are available from the corresponding author upon request.
